# Construction of Economic Data Management System Based on BP Neural Network

**DOI:** 10.1155/2022/9036917

**Published:** 2022-07-08

**Authors:** Xing Han

**Affiliations:** School of Economics, Harbin Normal University, Harbin 150025, Heilongjiang, China

## Abstract

In order to further understand the economic data management system and technology, in-depth research was conducted in the state of people's nervous system feeling. The method of building open platform algorithm to optimize and modify weight rule 2BP grid construction was used to study. According to the basic principle, the BP neural network which is more suitable for economic data management system was constructed. At the same time, to construct economic database resources, neural network system was mainly to simplify and abstract or simulate the human brain nervous system, which is not completely the same, but can also map the basic characteristics of many functions of the human brain. Through the analysis of the economic data of the neural network, the neural network is widely used in the economic data management, which not only improves the management level of enterprises, but also improves the benefits and profits of enterprises. Besides, it has application effect in predicting economic early warning risk analysis cost control strategy management enterprise credit evaluation and enterprise competitiveness evaluation.

## 1. Introduction

Artificial neural network is often called ANN for short, and it mainly needs to have a deep understanding of the human brain structure and operation mechanism, and build the simulator structure and intelligent behavior based on this theory. Artificial neural network is an engineering system. The first mathematical model of artificial neural network was put forward by psychologist McCulloch and mathematician Pitts in the early 1940s. It was also from this time that more researchers began to join in the research of neuroscience theory, and it also entered the era of theoretical research of neuroscience. Many researchers such as Rosenblatt F, Widrow, Klopf, and Hopfield J, followed by a long time of research and exploration, put forward the perception model. Perception model has the following characteristics: first is adaptability. It has powerful learning algorithms and self-organizing rules, which means it can adapt to any requirements in a constantly changing environment. Second is nonlinear processing. This perceptual model has the ability to perform pre-emptive tasks, but also has the ability to remove noise, which makes it better applied to classification and prediction problems. Third is parallel processing. The perceptual model has a structure of a large number of widely interconnected processing units, which also provides parallel processing and parallel distributed information storage capabilities.  Figure 1 shows the structure diagram of BP neural network. Among artificial neural networks, one of the most important models is BP (back propagation) neural network model, which is also widely used in various industries, such as data compression and classification. In simple terms, the BP neural network can be regarded as a mapping response, mapping the input to the output, and then the mapping is a highly nonlinear mapping.

## 2. Literature Review

Hu held that neural network system is a very complicated nonlinear dynamic system which is widely interconnected by neurons. Neural network system consists of a large number of processing units with very simple structure and function [1]. Duan reckoned that the neural network system is mainly to simplify and abstract or simulate the human brain nervous system, which is not completely the same, but can also map the basic features of many functions of the human brain. This is the current research level of brain nerve and intelligent excitation, and the technical level of VLSI can achieve the results and is also the basis of the current stage of neural network research [2]. Gupta and Singh studied that the basic common characteristic of neural network is nonlinear system, but there are other unique characteristics of its own, such as extensive interconnection among high-dimensional neurons, self-adaptability, and self-organization parallel processing characteristics [3]. Wu et al. found that in the process of generating dynamics, neural network system includes two aspects: one is the calculation process of neural network, and the other is the learning process of neural network [4]. Ahmed held that the computation process of neural network refers to the change process of mode in the active state of neural network system. The neural network enters into a certain state under the influence of input and is affected by the extensive interconnection between neurons and the dynamic nature of the neural network itself, leading to the rapid change of the excitation mode when the outside world stimulates it and then enters into a balanced state. Short-term memory is also based on this. The principle is to map a set of neighboring input states to the same equilibrium state [5]. Patil held that learning is the main method for neural networks to perform better computations. In the process of neural network learning, the intensity of interconnections between neurons will be affected by environmental information, and there will be certain changes. In this way, environmental information will be gradually stored in neural network, so as to establish long-term memory [6]. Kasimand Nugraha held that the learning process is mainly to build a self-organizing system and the environment to form a certain interaction structure, which can also help to acquire knowledge from the outside and then carry out corresponding learning [7]. Kasper held that the research on neural network theory can be divided into two modes at present: one is the learning neural network mode, and the other is the self-organization mode. In the process of the learning neural network mode, the calculation process is generally separated from the learning process, and the calculation process can be regarded as an autonomous dynamic process [8]. Strohmeier found that the process of research learning can be thought of as a systematic adjustment of the link strength of a neural network using an additional. However, because the organization mode is completely different from the learning neural network model, the organization mode of self-organizing neural network is generally in the learning process and calculation process, and has a certain correlation, and its connection strength as a dynamic system is variable [9]. Agarwal held that through continuous interaction of external environment, the purpose of self-organization can be achieved, and certain experience and relevant knowledge can be accumulated. Based on this self-organization, the system can constantly adjust and modify its own knowledge and experience, and modify the knowledge codes in the neural network [10].

## 3. Research Method

### 3.1. Build an Open Platform

Government units need to set up a more open platform, in order to increase the functions of the system at any time, and need to effectively use more standard product interface. In addition, in order to meet the requirements of the increased functionality of the system, the content types of various functions need to be implemented through relevant deployment [11]. Secondly, in order to reduce the complexity of economic data management and make it more easy and convenient to be operated in the practical operation, in the process of the construction of the system, it needs to reduce the complexity of the system construction. This is also largely a matter of staff operation, and it also addresses the problem of differences in the use of computer technology by business people across enterprises. This can facilitate the system in the actual operation of the management work and is more simple and easy to learn, and its content is easy to maintain. And this kind of operation platform operation needs a relatively more simple and easy to use human-computer interaction interface, which requires not only to follow the current advanced pace of system development, but also to meet the various requirements of the enterprise for site management and update. Thirdly, enterprises and public institutions need to set up a relatively open platform, so as to ensure that the management work is more targeted, but also promote the personalized submission of information. Only in this way can the internal staff of the enterprise master the data information, mobilize the enthusiasm of information production, and improve the work efficiency and quality [12]. The following formula is needed in the meantime:

(1) $$\begin{array}{c} W_{k}=W_{K}+\eta \cdot \left(\frac{-E}{\omega k}\right). \end{array}$$

### 3.2. Optimum of Algorithm

The meaning of the BP algorithm is to transform the complex input or output problem into a nonlinear optimization problem, that is, to take the network connection weight W as a variable and the error function as a target of a multivariate minimum problem [13]. In the specific process of BP algorithm, two steps are needed: the first is to use learning samples and network connection layer weights, in accordance with the order of input layer, hidden layer, and output layer, and check the output to each layer point; the second is to calculate in the opposite direction of the order, calculate the output deviation from the actual output, then form the error function, and then apply gradient descent to adjust the network weight, so as to reduce the error function [14]. These two steps need to be used alternately until convergence is shown. From the current stage of development, in the process of practical application of artificial neural network, most of the neural network models will use BP network or the form evolved from BP network in the process of practical construction [15]. Under the influence of the application of BP neural network, this paper focuses on how to apply BP neural network more effectively in the construction process of economic data management system, and puts forward a series of implementation procedures according to the actual situation, which has a certain guiding effect on the specific work and helps the staff to work smoothly. The existing neurons in neural network are generally divided into three types: input unit, hidden unit, and output unit [16]. The input unit generally obtains information through the external environment, while the output unit mainly transmits the information inside the neuron to the external environment. The implicit unit does not have a direct connection with the external environment, but it also plays an essential role and significance in the neural network. The input of a neuron *U*_*i*_(*i*=1,2,…, *m*) is the output of other neurons *O*_*k*_(*k*=1,2,…, *n*), and all the outputs need to be multiplied by their weights *W*_*ik*_, so that the total input *U*_*i*_ of the assembly can be obtained. In the meantime, formulas need to be applied:

(2) $$\begin{array}{c} {\text{net}}_{i}=\sum_{i=1}^{n}WikO_{k}. \end{array}$$

Among them, the interconnection structure of neural network system can be represented by matrix *W*, and the independent variables can be represented by *a*_*i*_ and net_*i*_. Select the active rule function *F*, so that the next active value can be generated, then *a*_*i*_(*t*+1) is chosen as an independent variable, and select a certain function *f* as the output function of the *U*_*i*_. *f* generally selects a certain threshold function, because only when the activity value of a neuron exceeds a certain threshold value, it can exert certain effects on its adjacent units. In the meantime, formulas need to be applied:

(3) $$\begin{array}{c} a_{i}\left(t+1\right)=F\left(a_{i}\left(t\right),{\text{net}}_{i}\right),\\ a_{i}\left(t\right)=F\left(a_{i}\left(t-1\right),{\text{net}}_{i}\left(t-1\right)\right). \end{array}$$

The composition of the neural network system is generally connected by many neurons, which can only reflect the structure of the neural network and also reflect the basic conditions of the neural network [17]. When researchers first studied the structure of neural network, it was only a relatively simple consisting of an input layer composed of input units unit and output layer composed of output unit. However, this kind of structure is relatively simple, so the ability of the neural network expressed by it is also limited to a certain extent. Through in-depth understanding and analysis of researchers, the hidden layer composed of hidden elements is finally introduced, thus forming a relatively common three-layer neural network model. This network model has a wide range of capabilities, and its application is not limited. It can be mapped to any function, which greatly improves the capability of neural networks [18].

### 3.3. Modify Weight Rules

Learning algorithms generally refer to the modification of weight rules in neural networks. From the current stage of development, people have developed unsupervised learning algorithms, which can automatically model structures from the environment, enhanced signal learning algorithms for multi-level network models, and error correction algorithms for solving hierarchical network learning. In the process of computation, neural network can be divided into two modes: one is serial mode, and the other is parallel mode. Serial operation mode refers to that when the neural network performs computation operation, only one neural unit's state is changed in each step; otherwise, it is parallel operation mode. In a word, the description of neurons can be started from as many as ten aspects, such as nerve cell, external environment, the state of a neural network, stable state, propagating rules, active rules, output function, interconnection model, learning algorithm, and operation mode. Through the unremitting efforts of many researchers, more than 30 neural network models have been constructed according to the basic neural network in half a century, laying a solid foundation for the subsequent research and development. The neural network system wants to find certain rules and features directly from the data, usually through training to achieve this purpose, which can also help to complete the mapping of arbitrary complex functions. It is this learning process that allows neural networks to be analyzed and modeled, and this process is like a black box in this way; neither model structure design nor parameter estimation is required. Nevertheless, it can still obtain good results through data-driven without input mode to verify information in advance. In neural network, the biggest advantage of learning process is more convenient and has certain plasticity [19]. Besides, the overall structure of the neural network does not require any adjustments or changes, the purpose of arbitrary relation learning can be realized only by some adjustment of weights, and then the changing state of the external environment can be accurately adapted and followed through progressive supplementary training samples [20]. Because of this, the working mode of neural network can realize the purpose of real time and self-adaptability.

#### 3.3.1. BP Grid Design

In the process of neural network work, information processing and storage are completed at the same time. Information has certain hidden characteristics, it has certain regularity in the distribution of neuron states and weights, and the main characteristic in this process is redundancy. If there is incomplete information or noisy information input, the neural network system can carry on certain association according to the distributed memory function of the information, so as to recover all the information.  Figure 2 shows the classification of neural network algorithms. At the same time, one of the most outstanding advantages of combining information processing and storage is to fundamentally eliminate the bottleneck effect between software and algorithm, which lays a solid foundation for achieving high-speed information processing. Neural network system is a powerful nonlinear dynamic system whose structure is characterized by high-dimensional and high-precision parallel computing [21]. It is the spectator activities of various neurons that build the macroscopic effect of the neural network system as a whole. It is this ability that enables neural networks to process high-risk data online and in real time. From the current stage of development, there are many models of artificial neural network, among which the error reversal propagation learning algorithm model, referred to as BP network, is the most widely promoted and applied. A typical BP network has three layers: the input layer and the hidden layer (also known as the middle layer, usually consisting of one layer or multiple layers) and the output layer. See Figure 3. BP network has many characteristics that other models do not have, among which the most prominent point is that error signals can be transmitted in reverse during the forward transmission of input signals. The input signal is usually to forward transfer of signals, according to certain rules or input layer ⟶ hidden layer ⟶ output layer, this time the network parameters (weights and threshold) will not change, each layer of neuron state will only correspond to the next level of neurons, and there is no correlation between the neurons in the same level. However, if the desired output signal cannot be obtained at the output layer, reverse transmission will be carried out; that is, the error signal of the network (the mean square error of the actual output and the expected output) will be transmitted in the opposite direction, that is, the output layer ⟶ hidden layer ⟶ input layer. In the process of reverse transmission of error signals, network parameters need to be adjusted and corrected, and the adjusted and corrected parameters will be used as the new parameters of the next set of input signals. In the working process of BP network, forward transmission of input signal and reverse transmission of error signal need to work alternately, and finally a set of network parameters can be obtained, so that the error between the actual output and the expected output can be within the range of standard error [22]. And according to relevant investigations and studies, there is a hidden layer in the neural network, and the hidden layer contains a sufficient number of neurons, so that any function can be approximated with arbitrary precision. Under the influence of BP neural network system, in order to better build economic data management system and analyze and explore the application of BP neural network in economic research, it is necessary to use related software for programming and calculation. The three specific application fields are shown in Figure 4.

#### 3.3.2. The BP Grid Construction

In the process of constructing BP network, it is necessary to determine the number of network input layer and output layer units and the number of hidden layer and the number of units in each hidden layer initial weight and other important data. Research scholar has proved through a large number of studies that for any continuous function in a closed interval, it can be approximated by a single hidden layer feedforward network. In other words, a feedforward network with a single hidden layer can complete any larger and more complex function, but this does not mean that the BP network with a single hidden layer is the best, which needs to be judged according to the actual situation. Because when the number of hidden layers is increased, the expression ability of BP network can be effectively enhanced. But it also has a disadvantage, that is, it will have a certain impact on the convergence speed. Therefore, in the specific process of applying BP network, it is necessary to judge according to the actual situation and determine the specific purpose of the number of hidden layers, so as to give full play to the greatest advantage of BP network [23]. Experimental methods can be used to determine the number of hidden layers. The basic principle of determining the number is that the number of hidden layers selected should be as small as possible on the basis of reflecting the input and output relationship, so as to ensure the simple network structure. In the process of testing, if it is found that there are a large number of units in a single hidden layer, the single hidden layer can be transformed into a double hidden layer. During this period, the formula needs to be applied:

(4) $$\begin{array}{c} n1=\sqrt{n+m}+a, \end{array}$$

(5) $$\begin{array}{c} n1=\;\log_{2}\;n. \end{array}$$

*m* is the number of output neurons, *n* is the number of input neurons, and *a* is a constant *L* between 1–10. Although the basic principles of BP network construction have been formulated, it is necessary to conduct research and analysis based on the actual situation in the specific construction process. In order to ensure that the system network can achieve better prediction effect and, at the same time in the normal operation of the system convergence speed, eliminate the dimension, the first step to do is to normalize the input data. Adjust the data to a certain extent to the range of [0.1, 0.9] so as to make the *S* function change in between. The recent trend of neural network economic data is shown in Figure 5 and the performance capability of the BP neural network in Figure 6. In addition, the change gradient is obvious, which can reduce the convergence time of the network to some extent and improve the performance of the system, as shown in Figure 7; during this period, the formula needs to be applied:

(6) $$\begin{array}{c} x^{\prime }=0.1+\frac{0.8\left(x-x_{\min}\right)}{x_{\max}-x_{\min}}. \end{array}$$

*x* represents the initial data, *x*_max_ represents the maximum value in the initial data, *x*_min_ represents the minimum value in the initial data, and *x*′ represents the normalized data.

According to the algorithm flow mentioned in the previous article, the corresponding software is used to program, and the normalized data are used to train the BP network. In terms of the selection of functions, tansig-type transfer function is used for the hidden layer, and Logsig-type transfer function is used for the output layer to continuously modify and adjust according to the actual situation. Finally, the number of hidden layers of the BP network is determined as 6. In order to better optimize and improve the network, the gradient descent algorithm (VLBP) with variable learning rate is generally used in this process, so that the learning rate can be adjusted according to the change of the error [24]. When the error gradually decreases and is closer to the standard accuracy, it indicates that the correction direction is correct. However, if the error increases and exceeds the pre-set value, it indicates that the correction is excessive, which will cause the learning rate to decline. By using VLBP algorithm, when traingdx is used as the training function, the learning rate is set at 0.05, then the growth ratio of the learning rate is 1.04, and the decline ratio is 0.8. During this period, the formula needs to be applied:

(7) $$\begin{array}{c} \eta \left(q+1\right)\left\{\begin{array}{cc} 1.04\eta \left(q\right), & E\left(q+1\right)<E\left(q\right),\\ 0.8\eta \cdot 8\eta , & E\left(q+1\right)<E\left(q\right). \end{array}\right. \end{array}$$

After the network training, the errors and network output results can be statistically analyzed as a whole according to the actual training situation, and corresponding charts can be drawn, as shown in Figures 8 and 9.

According to the curve shown in Figure 6, it is not difficult to see that the error of network training decreases gradually with the increase of the number of iterations, and there is an inverse relationship between the two. After 4000 iterations, the error value of network is between 4.0798*E* − 0.05 [25].

According to the curve shown in Figure 7, the solid line is the fitting curve obtained, and *∗* represents the actual data in the training process. It can be seen from Figure 7 that the BP network wants to control the error value within the minimum range, and the output result is basically consistent with the real value of the training sample [26]. In the process of comparing BP network and regression equation, it is necessary to apply formula (6) to conduct statistical analysis on the data from 2000 to 2003 and conduct in-depth study according to BP network. The study shows that the economic variables studied are the same, so this study has certain comparability, as shown in Table 1.

(8) $$\begin{array}{c} Y=0.449X^{0.464}. \end{array}$$

It can be seen from Table 1 that BP neural network fits economic data very accurately. Although the calculation results of regression equation can also reflect the specific situation of economic data and economic development trend, the accuracy of its fitting results is obviously not as high as that of BP neural network [27].

## 4. Result and Analysis

With the continuous development of China's economy, enterprises and institutions pay more attention to the statistics of economic data in the process of development. Therefore, extracting data with greater application value from a large number of data resources plays a guiding role in the economic development planning and major decisions of enterprises and institutions. Generally starting from the financial transaction center and asset management, centralized data collation and effective use of the collated data can promote economic development.

The economic data management system based on BP neural network constructs a black box processing mode. In this process, it only needs to input sample data to train the network after determining the network parameters, without considering the functional relationship between economic variables. The algorithm principle and self-learning feature of the BP network enable it to fully dig out the regularity hidden in the sample data, realize the nonlinear mapping from input space to output space, and accurately fit the sample data [28]. First of all, the computer should be used to initialize the network and set a set of initial weights according to the corresponding situation. Secondly, a group of sample data is randomly selected and the network is trained to calculate the neuron output of the hidden layer and the output layer according to the trained data. At the same time, the error data between the actual output and the expected output should also be calculated. The error accuracy is shown in Figure 10. And the error signal is in accordance with the output layer ⟶ hidden layer ⟶ input layer in the order of reverse transmission, after repeated continuous alternating operation, so that the error between the actual output and the expected output can gradually be reduced as shown in Figures 11 and 12. When the error data reach the standard accuracy, the training can be stopped; if the error data do not reach the standard accuracy, continuous training is required until the error data reach the standard accuracy [29].

## 5. Conclusion

BP neural network is widely used in economic data management, improves the management level of enterprises, and improves the benefits and profits of enterprises. It has application effect in predicting economic early warning risk analysis, cost control strategy management, enterprise credit evaluation, and enterprise competitiveness evaluation. In the implementation process, the selection of the number of hidden layers, the selection of the number of hidden layer units, and the processing of data need to be analyzed according to the actual situation, so as to build a neural network with good stability, high accuracy, and fast operation speed in the experiment. In this process, relevant personnel can use more advanced, mature, stable, and scientific and technological means that meet relevant standards to constantly supplement and increase the functions of the system. Finally, in order to control the flow of information, users need to apply relevant workflow technology according to the actual situation, which is more conducive to the organizational structure of the enterprise, based on the role of the staff working authority and flexible workflow settings. In view of the above series of situations, the construction of economic data management system is of great significance. Firstly, it can help related enterprises and institutions of various professional systems for exterior performance presentation logic and information processing are relatively separated, so that we can let the professional skills of the staff working in their jobs and can also be on the basis of economic data management system to help the staff to achieve the coordination of all work. This also helps to provide more secure spaces for personal use and also helps to establish a database that is more suitable for the work of each department to archive the economic data generated in operations and production.

## Figures and Tables

**Figure 1:** BP neural network structure diagram.

**Figure 2:** Neural network algorithm classification.

**Figure 3:** Three layers of the BP network.

**Figure 4:** Three application fields of neural network.

**Figure 5:** Recent trends in neural network economic data.

**Figure 6:** BP network presentation ability.

**Figure 7:** Initial data versus altered data.

**Figure 8:** Training error curve.

**Figure 9:** Network output.

**Figure 10:** Accuracy of data error.

**Figure 11:** Input layer reverse transfer speed.

**Figure 12:** Output layer reverse transfer speed.

**Table 1:** Fitting results of BP neural network and regression equation.

Year	Actual value (%)	Regression equation results (%)	Error information	BP neural network result (%)	Error information
2000	27.5	27.5	0.0	27.3	−0.2
2001	27.7	28.5	0.8	28.1	0.4
2002	28.6	29.4	0.8	28.3	−0.3
2003	29.3	30.9	1.6	29.3	0.0

## Data Availability

No data were used to support this study.
